# Establishment of a rapid and footprint-free protocol for differentiation of human embryonic stem cells into pancreatic endocrine cells with synthetic mRNAs encoding transcription factors

**DOI:** 10.1186/s13287-018-1038-3

**Published:** 2018-10-25

**Authors:** Hideomi Ida, Tomohiko Akiyama, Keiichiro Ishiguro, Sravan K. Goparaju, Yuhki Nakatake, Nana Chikazawa-Nohtomi, Saeko Sato, Hiromi Kimura, Yukihiro Yokoyama, Masato Nagino, Minoru S. H. Ko, Shigeru B. H. Ko

**Affiliations:** 1 Department of Systems Medicine, Keio University School of Medicine, 35 Shinanomachi, Shinjuku, Tokyo, 160-8582 Japan; 2 Division of Surgical Oncology, Department of Surgery, Nagoya University Graduate School of Medicine, Nagoya, Aichi Japan

**Keywords:** Embryonic stem cells, Endocrine differentiation, Transcription factors, Synthetic mRNAs, Pancreatic β cells, PDX1, NKX6.1, siPOU5F1

## Abstract

**Background:**

Transplantation of pancreatic β cells generated in vitro from pluripotent stem cells (hPSCs) such as embryonic stem cells (ESCs) or induced pluripotent stem cells (iPSCs) has been proposed as an alternative therapy for diabetes. Though many differentiation protocols have been developed for this purpose, lentivirus-mediated forced expression of transcription factors (TF)—PDX1 and NKX6.1—has been at the forefront for its relatively fast and straightforward approach. However, considering that such cells will be used for therapeutic purposes in the future, it is desirable to develop a procedure that does not leave any footprint on the genome, as any changes of DNAs could potentially be a source of unintended, concerning effects such as tumorigenicity. In this study, we attempted to establish a novel protocol for rapid and footprint-free hESC differentiation into a pancreatic endocrine lineage by using synthetic mRNAs (synRNAs) encoding *PDX1* and *NKX6.1*. We also tested whether *siPOU5F1*, which reduces the expression of pluripotency gene POU5F1 (also known as OCT4), can enhance differentiation as reported previously for mesoderm and endoderm lineages.

**Methods:**

synRNA-*PDX1* and synRNA-*NKX6.1* were synthesized in vitro and were transfected five times to hESCs with a lipofection reagent in a modified differentiation culture condition. *siPOU5F1* was included only in the first transfection. Subsequently, cells were seeded onto a low attachment plate and aggregated by an orbital shaker. At day 13, the degree of differentiation was assessed by quantitative RT-PCR (qRT-PCR) and immunohistochemistry for endocrine hormones such as insulin, glucagon, and somatostatin.

**Results:**

Both PDX1 and NKX6.1 expression were detected in cells co-transfected with synRNA-*PDX1* and synRNA-*NKX6.1* at day 3. Expression levels of insulin in the transfected cells at day 13 were 450 times and 14 times higher by qRT-PCR compared to the levels at day 0 and in cells cultured without synRNA transfection, respectively. Immunohistochemically, pancreatic endocrine hormones were not detected in cells cultured without synRNA transfection but were highly expressed in cells transfected with synRNA-*PDX1*, synRNA-*NKX6.1*, and *siPOU5F1* at as early as day 13.

**Conclusions:**

In this study, we report a novel protocol for rapid and footprint-free differentiation of hESCs to endocrine cells.

## Background

Type 1 diabetes mellitus (T1DM) is an endocrine disorder that is characterized by autoimmune destruction of insulin-producing β cells. To treat T1DM patients, the primary therapy is injections of exogenous insulin to control their blood glucose levels throughout their lives. However, they often suffer from diabetic complications such as cardiovascular or cerebrovascular disturbance, retinopathy, kidney failure, and neuropathy that lead to an impaired quality of life. An alternative therapy is homologous pancreatic islet transplantation. However, the application of this therapy is limited because of the shortage of donor islets and the requirement of lifelong immunosuppression therapy after transplantation. To overcome these obstacles, the use of pancreatic β cells differentiated in vitro from human embryonic stem cells (ESCs) or induced pluripotent stem cells (iPSCs) has been proposed [1–7]. However, these differentiation protocols require a rather long period of time and complicated culture steps, posing further challenges for their clinical application.

PDX1 and NKX6.1 are well-known transcription factors (TFs) for endocrine cell development. PDX1 (pancreatic and duodenal homeobox-1) is expressed in foregut endoderm and plays a pivotal role in the differentiation of all pancreatic cell types, because the entire pancreas is absent in PDX1 knockout mice at birth [8]. NKX6.1 (NK6 homeobox-1) is expressed in pancreatic endoderm and endocrine precursor cells and is essential for β cell identity, controlling cell lineages between endocrine and acinar cell fate [9–11]. It has also been demonstrated that iPSCs can be differentiated into mature insulin-producing cells by lentivirus-mediated overexpression of PDX1 and NKX6.1 using the Tet-On System combined with endocrine differentiation medium [12]. This study showed that PDX1 and NKX6.1 are crucial factors for differentiating hPSCs into insulin-producing endocrine cells.

Previously, we have reported a novel differentiation method for hESCs and hiPSCs into neuronal cells [13], skeletal muscle cells [14], and epithelial cells [15] by introducing synthetic mRNAs (synRNAs) encoding transcription factors specific to the targeted differentiated cells. Differentiation by synRNAs holds many desirable features for further clinical application, because it allows rapid, efficient, and footprint-free differentiation of human pluripotent stem cells [16]. We have also reported that the forced silencing of pluripotency master regulator POU5F1 (also known as OCT4, OCT3/4) by *siPOU5F1* facilitates synRNA-based hPSC differentiation [17].

In this study, we aimed to establish a rapid, footprint-free, and simpler differentiation protocol for hESCs into pancreatic endocrine cells, especially insulin-producing β cell-like cells, by the combined introduction of synRNAs encoding *PDX1*, *NKX6.1*, and *siPOU5F1*.

## Methods

### Cells and culture media

SEES-3 human ES cells were obtained from the National Center for Child Health and Development, Japan [18], and cultured under feeder-free conditions in StemFit AK02N medium (Ajinomoto, Tokyo, Japan) on laminin511 E8 fragment (iMatrix-511: Nippi, Tokyo, Japan)-coated dishes. All experiments were performed in accordance with the Guidelines for Derivation and Utilization of Human Embryonic Stem Cells by the Ministry of Education, Culture, Sports, Science, and Technology, Japan. Experimental protocols were approved by the Ethics Committee of Keio University School of Medicine for human stem cell experiments (No. 2012-01) and for recombinant DNA experiments (No. 24-010-12).

### Modified RNA synthesis and siRNA

The open reading frames for PDX1 and NKX6.1 were subcloned into a pCRII construct containing the 5′ and 3′ untranslated regions of mouse alpha-globin to prepare the templates used for synthesizing the mRNAs. The modified mRNAs were produced as described previously [19]. *siPOU5F1* (silencer Select ID s10873) was obtained from Life Technologies.

### In vitro differentiation of human ES cells

SEES-3 human ES cells were seeded and cultured on 24-well plates coated with 1:30 diluted Matrigel (Corning, NY) at a density of 8.0 × 10^4^ cells per well in StemFit AK02N medium with 10 μM Y-27632 (WAKO, Japan) for 2 days. At ~ 80% confluency, *PDX1* and *NKX6.1* synthetic-mRNA (synRNA) introduction was started. mRNAs encoding these transcription factors were transfected with Lipofectamine MessengerMax Transfection Reagent (Thermo Fisher Scientific, MA) every 12 h (total of five times) according to the manufacturer’s instructions. For POU5F1 silencing, *siPOU5F1* was transfected once and was included only in the first cocktail of *PDX1* and *NKX6.1* mRNA transfection. A total of 1 μg mRNA in opti-MEM-reduced serum media (Thermo Fisher Scientific) was mixed with 2 μl MessengerMax Reagent in Opti-MEM media and incubated for 5 min at room temperature. B18R interferon inhibitor (eBioscience) was included in the transfection complex to inhibit the interferon response caused by mRNA introduction to the cells. The differentiation medium was replaced 3 h after every transfection.

We replaced the differentiation medium every 12 h for 3 days; the process is described as d*X*-a (first medium change on day *X*) to d*X*-b (second medium change on day *X*). The differentiation conditions used were as follows: d0-a: RPMI 1640 medium (Thermo Fisher Scientific) supplemented with 1:100 B27 (Thermo Fisher Scientific), 1:5000 ITS (Thermo Fisher Scientific), 100 ng/ml activin A (R&D Systems, MN), and rhWNT3a (R&D Systems, MN); d0-b: RPMI 1640 medium supplemented with 1:100 B27, 1:2000 ITS, and 100 ng/ml activin A; d1-a: RPMI 1640 medium supplemented with 1:100 B27, 1:1000 ITS, 2.5 μM TGFbi IV (Merck KGaA, Germany), and 25 ng/ml KGF (PeproTech, NJ); d1-b: RPMI 1640 medium supplemented with 1:100 B27, 1:1000 ITS, and 25 ng/ml KGF; d2-a: DMEM (nacalai tesque, Japan) with 25 mM glucose supplemented with 1:100 B27 and 3 nM TTNBP (Sigma-Aldrich, Germany); d2-b: DMEM with 25 mM glucose supplemented with 1:100 B27, 50 ng/ml EGF (PeproTech), 50 ng/ml KGF, and 3 nM TTNBP. Twelve hours after the last transfection, cells were dissociated into single cells by incubation with TrypLE (Thermo Fisher Scientific). Cells were counted and seeded on 24-well low-binding plates at a density of 1.6 × 10^5^ cells per well in 500 μl d3–7 medium supplemented with 10 μm Y-27632 and 10 ng/ml heregulin-b1(PeproTech). Plates were placed on an orbital shaker at 100 rpm for the rest of the culture period, d3–7: DMEM with 25 mM glucose supplemented with 1:100 B27, 500 nM LDN193189 (Stemgent, MA), 3 nM TBP (Calbiochem), 1000 nM ALKi II (Cayman Chemical, MI), and 25 ng/ml KGF. From days 3 to 7, medium was replaced every 2 days by removing 250 μl of medium and adding fresh 250 μl of medium. After culturing for 5 days, the medium was then changed to d8–12 medium, d8–12: DMEM with 2.8 mM glucose supplemented with 1:100 Glutamax (Gibco) and 1:100 NEAA (nacalai tesque).

### Immunocytochemistry

After removing the culture medium, cells were rinsed with PBS once and fixed with 4% paraformaldehyde (Wako, Japan) for 10 min at room temperature and blocked with 0.3% Triton-X-100 (Sigma-Aldrich, Germany) and 5% BSA in PBS for 30 min at room temperature. The fixed cells were then incubated with primary antibodies overnight at 4 °C. The primary antibodies used were as follows: goat anti-PDX1 (1:100; R&D Systems, AF2419), mouse anti-NKX6.1 (1:50; DSHB, F55A10-s), goat anti-FOXA2 (1:100; R&D Systems, AF2400), mouse anti-HNF1B (1:100; Sigma-Aldrich, HPA002083), goat anti-HNF4A (1:100; Santa Cruz, sc-6556), rabbit anti-HNF6 (1:100; Santa Cruz, sc-13050), and mouse anti-NEUROD1 (1:100; Abcam, ab60704). After washing with PBS three times, cells were incubated for 60 to 120 min at room temperature with Alexa Fluor conjugated secondary antibodies (1:1000; Life Technologies). After washing with PBS twice, DAPI (1:1000; Life Technologies) with PBS was added to stain the nucleus. Images were captured using an Olympus microscope IX73.

### Immunocytochemistry for cryosections

After washing with PBS once, cell clusters were fixed with 4% paraformaldehyde (PFA) overnight at 4 °C. Following fixation, PFA was removed and cells were washed three times with PBS for 5 min each and equilibrated in 30% sucrose solution overnight at 4 °C. The cells were overlaid with OCT Compound and frozen using liquid nitrogen. The frozen blocks were sectioned at 10 μm. The sections were washed with PBS twice for 5 min each and blocked with 0.3% Triton-X-100 and 5% BSA in PBS for 1 h at room temperature. Primary antibodies were added overnight at 4 °C in a blocking buffer. After washing with PBS three times for 5 min, secondary antibodies were added for 30 min at room temperature in a blocking buffer. After washing with PBS three times for 5 min, sections were mounted with VECTASHIELD Mounting Medium with DAPI (Vector Laboratories) on glass slides.

### Quantitative RT-PCR

Total RNA was extracted from cells using TRIzol Reagent (Thermo Fisher Scientific) and Direct-Zol RNA Miniprep (ZYMO RESEARCH) according to the manufacturer’s instructions. Quantitative RT-PCR (qRT-PCR) was performed using SYBR Fast qPCR Mix (Takara Bio, Japan) and Thermal Cycler Dice Real Time System III (Takara Bio). The Ct values and relative expression levels were normalized by glyceraldehyde-3-phosphate dehydrogenase (*GAPDH*) levels.

### Statistical analysis

The difference between samples was compared by the two-tailed Student’s *t* test and statistical significance was considered as *p* < 0.05. All data were presented as mean ± SEM (standard error of the mean).

## Results

### Production and test of synRNAs

Generation of synthetic mRNA (synRNAs) was performed as reported previously (Fig. 1a) [13]. To evaluate the co-transfection efficiency of synRNAs to hESCs, we co-transfected synRNAs encoding green fluorescence protein variants—Emerald (green) and mCherry (red)—and monitored the protein expression by microscopy 8 h after transfection. Each fluorescent protein was efficiently expressed and the expressions of two proteins were clearly merged in most cells (Fig. 1b). This result confirmed the high efficiency of the synRNA-based protein expression in hESCs.

**Fig. 1:** The efficiency of synthetic mRNA transfection of *PDX1* and *NKX6.1* into SEES3 human ESCs. **a** Generation of synthetic messenger RNAs. ARCA: anti-reverse cap analog, pseudo-UTP: pseudouridine-5′-triphosphate, 5-Me-CTP: 5-methyl cytidine-5′-triphosphate. **b** Expression of synthetic messenger RNA for fluorescent proteins Emerald and mCherry in SEES3 human ESCs. Scale bars, 200 μm

### Generation of PDX1^+^/NKX6.1^+^ pancreatic endoderm/endocrine precursor cells

As a first step to establish a differentiation protocol, we started with the protocol reported by Russ et al. [3], because their method is simple and rapid compared with other protocols for the differentiation of hPSCs into insulin-producing cells. We noticed that the protocol takes 7–9 days until PDX1^+^ or PDX1^+^/NKX6.1^+^ cells appear, and additional 3 weeks until insulin^+^ β-like cells appear. Therefore, we first focused on generating PDX1- and NKX6.1-positive pancreatic endoderm cells by exogenously introducing synRNA-*PDX1* and synRNA-*NKX6.1* together with *siPOU5F1* with their pancreatic endocrine differentiating conditions (Fig. 2a).

**Fig. 2:** Schematic of differentiation protocol and characterization at day 3. **a** The differentiation protocol for human ESCs into pancreatic endocrine cells. The transfection schedule, growth factor, small chemical molecules, medium, and duration for each stage are shown. **b** Gene expression of *PDX1* (*n* = 4) and *NKX6.1* (*n* = 6) was analyzed by qRT-PCR at day 3. The *Y* axis indicates the relative change of mRNA expression compared with that of ES and no transfection (=1). Results were shown relative to the endogenous control *GAPDH*. *P < 0.05. Error bars represent SEM (*n* = 5). **c** Protein expression of PDX1 and NKX6.1 was analyzed by immunostaining at day 3. Scale bars, 50 μm

We analyzed the expression levels of PDX1 and NKX6.1 by qRT-PCR after five transfections and compared the results with those of day 0 (D 0) that is a cellular state of undifferentiated ES cells and cells treated with differentiation medium alone (no transfection). Using PCR-primers detecting both endogenous and exogenous PDX1 and NKX6.1, the expression levels of PDX1 increased 147-fold compared with that of no transfection. The expression of NKX6.1 increased 286-fold compared with that of no transfection (Fig. 2b), indicating that both PDX1 and NKX6.1 were significantly overexpressed in cells transfected with mRNAs encoding these transcription factors as early as at day 3. Although there was a significant difference in the expression levels between PDX1 and NKX6.1, this result may simply be a reflection of the difference of translation efficiency of *PDX1* and *NKX6.1* synRNAs in these cells.

Using antibodies against PDX1 and NKX6.1, protein expression was immunocytochemically confirmed: a significant number of PDX1^+^/NKX6.1^+^ cells were present even at day 3 (Fig. 2c). The ratio of PDX1^+^, NKX6.1^+^, and PDX1^+^/NKX6.1^+^ was 23%, 20%, and 16%, respectively. Taken together, these results indicated that hESCs were able to differentiate into pancreatic endoderm cells within 3 days with the aid of synRNA-*PDX1*, synRNA-*NKX6.1*, and *siPOU5F1*.

### Endoderm and endocrine precursor cell marker expression

To examine whether these PDX1^+^ and/or NKX6.1^+^ cells are indeed endoderm or endocrine precursor cells, marker gene expressions were analyzed by qRT-PCR at day 3 just after five consecutive transfections of synRNA-*PDX1* and synRNA-*NKX6.1* together with *siPOU5F1*.

The expression levels of definitive endoderm (DE) markers *FOXA2* and *SOX17* in cells with synRNA transfection were increased 300- and 4980-fold, respectively, compared with the level in ES cells. Although the expression level of *SOX17* showed no difference in cells with no transfection and synRNA-*PDX1*/synRNA-*NKX6.1*-transfected, the expression level of *FOXA2* in cells transfected with synRNAs was increased significantly compared with the level in cells with no transfection (Fig. 3a). FOXA2 protein expression was detected in cells transfected with synRNA-*PDX1*/synRNA-*NKX6.1* by immunocytochemical analysis. The number of FOXA2-positive cells in cells with no transfection and PDX1/NKX6.1 transfection was 13% and 94%, respectively (Fig. 3d), indicating that the introduction of synRNA-*PDX1*/synRNA-*NKX6.1* further promotes hESCs’ differentiation into DE.

**Fig. 3:** Expression levels of pancreatic transcription factors at day 4. **a** Definitive endoderm (DE): *FOXA2* (*n* = 5) and *SOX17* (*n* = 6). **b** Primitive gut tube (PG): *HNF1B* (*n* = 5), posterior foregut endoderm: *HNF6* (*n* = 6). **c** Pancreatic endoderm and endocrine precursor (PE): *NGN3* (*n* = 6), *PAX4* (*n* = 6), *NKX2.2* (*n* = 6), and *NEUROD1* (*n* = 6). Compared with ES, no transfection (=1) and transfection. *P < 0.05. N.S no significance. Error bars represent SEM (*n* = 5). **d** Immunofluorescence images of cells at day 3 for FOXA2, HNF1B, HNF4A, HNF6, and NEUROD1 all in green. Scale bars, 100 μm

The expression levels of primitive gut tube (PGT) markers *HNF1B* and *HNF4A* in cells with synRNA transfection was increased 2.4-fold and 16.5-fold, respectively, compared to cells with no transfection (Fig. 3b). Posterior foregut endoderm (PFE) marker—*HNF6*—was increased 1.5-fold compared with that of no transfection. Although the protein expression of HNF6 was not detected, we confirmed HNF4A and HNF1B protein expression in both no transfected cells and synRNA-transfected cells. The number of HNF4A-positive cells in cells with no transfection and synRNA-*PDX1/NKX6.1* transfection was 1.5% and 14.1%, and the number of HNF1B-positive cells was 28.2% and 13.4%, respectively (Fig. 3d). These results indicate that the introduction of synRNA-*PDX1*/synRNA-*NKX6.1* further promotes differentiation to PGT/PFE cells.

NEUROGENIN3 (NGN3), PAX4, NKX2.2, and NEUROD1 are markers of endocrine precursor (PE) cells. The expression levels of *NGN3*, *PAX4*, and *NKX2.2* in cells transfected with synRNA-*PDX1*/synRNA-*NKX6.1* were not increased significantly compared with that of no transfection. The other PE marker, *NEUROD1*, showed slight increase by qRT-PCR in cells transfected with synRNA-*PDX1*/synRNA-*NKX6.1* compared to the expression levels in cells treated with differentiation medium alone (Fig. 3c), but the protein expression of NEUROD1 was not detected by immunocytochemistry (Fig. 3d). These results may indicate that synRNA-*PDX1* and synRNA-*NKX6.1* and *siPOU5F1* transfection differentiate hESCs to cells in the PGT or PEE stage, but not to pancreatic endocrine precursor cells at day 3.

### PDX1^+^/NKX6.1^+^ cells further differentiate to pancreatic endocrine cells in three-dimensional culture conditions

Three-dimensional (3D) culture by cell aggregation is known to promote the maturation of cells in the pancreatic endocrine lineage [4]. To further promote differentiation to terminally differentiated insulin-positive β-like cells, PDX1^+^/NKX6.1^+^ cells were aggregated and cultured on an orbital shaker at 100 rpm from days 3 to 13. A few small buddings were observed at day 5 and cystic structures were observed at day 9 (data not shown) in cell clusters transfected with synRNA-*PDX1* and synRNA-*NKX6.1* (Fig. 4a, lower panels), but the cell clusters with culture conditions alone showed no morphological changes during the culture period to day 13 (Fig. 4a, upper panels).

**Fig. 4:** Characterization of pancreatic hormone in human ESC-derived culture at day 13. **a** Time course culture of non-transfected and transfected cells at days 5, 9, and 13. Scale bars, 500 μm. **b** Time course of gene expressions. Insulin, glucagon, and somatostatin were analyzed by qRT-PCR at day 13. The *Y* axis indicates the relative change of mRNA expression compared with that of no transfection. Results were shown relative to the endogenous control *GAPDH*. *P < 0.05. Error bars indicate SEM *n* = 4. **c** Upper panels show insulin (red) and glucagon (green) immunostainings and a DAPI staining (blue) at day 13. Scale bars, 200 μm. Lower panels show insulin (red), glucagon (green), and somatostatin (blue) immunostainings and a DAPI staining (gray) at day 13. Monohormonal insulin-positive cells: white arrow heads. Scale bars, 15 μm

To test whether these cells were indeed differentiated into pancreatic endocrine cells, we next examined the expression levels of pancreatic hormones—insulin, glucagon, and somatostatin—by qRT-PCR. In culture conditions alone (no transfection), insulin expression was increased in cells from days 6 to 13 compared with those at day 0 or day 3. In synRNA-transfected cells, insulin expression was significantly increased (approximately tenfold) compared with those in cells with no transfections after days 11 to 13, indicating that synRNA introduction to cells at days 0–2 promoted differentiation of cells to pancreatic endocrine cells at days 11–13. Glucagon expression was increased at days 11–13 and somatostatin expression was increased after day 6 in cells with no transfection compared with that of control cells, respectively. The introduction of synRNAs significantly increased glucagon and somatostatin expression (approximately tenfold) compared with cells with no transfection at days 11 and 13 (Fig. 4b). These results clearly indicated that in addition to pancreatic endocrine differentiation culture conditions, the introduction of synRNA-*PDX1*, synRNA-*NKX6.1*, and *siPOU5F1* to hESCs furthers and efficiently promotes endocrine differentiation.

To confirm the spatial expression pattern of pancreatic endocrine hormones in cell clusters, expression of insulin, glucagon, and somatostatin was immunohistochemically examined. Under pancreatic differentiation culture conditions with no mRNA transfection, expression of insulin and glucagon was not observed at day 13. However, we confirmed that cells expressing insulin and glucagon appeared in mRNA-transfected cells at day 13 (Fig. 4c). The ratio of the cells expressing insulin, glucagon, and somatostatin was 5.6%, 2.6%, and 3.4%, respectively. Notably, there are some monohormonal, insulin-positive, but glucagon- and somatostatin-negative cells (Fig. 4c, white arrow head) among pancreatic endocrine hormone-expressing cells with synRNA-*PDX1/NKX6.1* transfection.

## Discussion

In this study, we have established a rapid, efficient, and footprint-free protocol of hESC differentiation into pancreatic endocrine cells by introducing synRNA-*PDX1* and synRNA-*NKX6.1* together with *siPOU5F1*. By adding these synRNAs, the expression level of insulin-positive cells was increased about ten times compared to cells with no transfection, and insulin-positive cells appeared at as early as day 11 by qRT-PCR and at day 13 by immunohistochemical examinations. With the aid of transcription factor mRNA transfection, we were able to shorten the time required for the differentiation of pancreatic endocrine hormone-expressing cells for human ESCs.

The definitive endoderm is the first step to induce the differentiation of pancreatic endocrine cells from pluripotent stem cells. In previous studies by others, more than 2 weeks were necessary just to induce PDX1^+^/NKX6.1^+^ cells. We have previously reported differentiation methods for neurons [13], skeletal muscle cells [17], and lacrimal gland epithelium-like cells [15] in a short period of time by introducing synthetic mRNAs encoding specific transcription factors required for the target mature cells. In this study, we have attempted to shorten the period of time required for the induction of pancreatic endocrine cells from human pluripotent stem cells with the same differentiation method using *PDX1* and *NKX6.1* synthetic mRNAs. By introducing these transcription factors, it was possible to induce definitive endoderm and primitive gut tube marker-expressing cells within 3 days from hESCs.

Immunohistochemical examination confirmed the presence of pancreatic endocrine hormones such as insulin, glucagon, and somatostatin at day 13. Although most insulin-positive cells were glucagon-positive (double positive) and some of them were also somatostatin-positive (triple positive) cells, insulin-only-positive, monohormonal, so-called mature β cells were present at as early as day 13. Previous studies have shown the expression of NKX6.1 is required for the development of the β cell lineage from endocrine progenitors. Nostro et al. have identified the pathways that regulate the development of endocrine cells in vivo, and they found that NKX6.1 expression is a key factor to generate mature β cells [20]. Our study may also indicate the importance of NKX6.1^+^ expression for the development of monohormonal β cell differentiation from human pluripotent stem cells.

This RNA-based differentiation method has advantages over others for potential therapeutic applications, since it is footprint-free and integration-free to the host genome. Thus, our method may be well suited to producing pancreatic endocrine cells from pluripotent stem cells for future regenerative therapies for diabetes.

## Conclusion

By introducing synthetic mRNAs encoding two pancreatic transcription factors, *PDX1* and *NKX6.1* together with *siPOU5F1*, we were able to successfully establish a rapid and footprint-free protocol for differentiating pancreatic endocrine hormone-expressing cells from hESCs. With this protocol, HNF1B- and HNF4A-expressing primitive gut tubes were generated at day 3, and pancreatic hormone-expressing cells such as insulin, glucagon, and somatostatin were generated at as early as day 13.

## References

[1] Pagliuca FW, Millman JR, Gurtler M, Segel M, Van Dervort A, Ryu JH, Peterson QP, Greiner D, Melton DA (2014). Generation of functional human pancreatic beta cells in vitro. Cell.

[2] D'Amour KA, Bang AG, Eliazer S, Kelly OG, Agulnick AD, Smart NG, Moorman MA, Kroon E, Carpenter MK, Baetge EE (2006). Production of pancreatic hormone-expressing endocrine cells from human embryonic stem cells. Nat Biotechnol.

[3] Russ HA, Parent AV, Ringler JJ, Hennings TG, Nair GG, Shveygert M, Guo T, Puri S, Haataja L, Cirulli V (2015). Controlled induction of human pancreatic progenitors produces functional beta-like cells in vitro. EMBO J.

[4] Toyoda T, Mae S, Tanaka H, Kondo Y, Funato M, Hosokawa Y, Sudo T, Kawaguchi Y, Osafune K (2015). Cell aggregation optimizes the differentiation of human ESCs and iPSCs into pancreatic bud-like progenitor cells. Stem Cell Res.

[5] Saxena P, Heng BC, Bai P, Folcher M, Zulewski H, Fussenegger M (2016). A programmable synthetic lineage-control network that differentiates human IPSCs into glucose-sensitive insulin-secreting beta-like cells. Nat Commun.

[6] Rezania A, Bruin JE, Arora P, Rubin A, Batushansky I, Asadi A, O'Dwyer S, Quiskamp N, Mojibian M, Albrecht T (2014). Reversal of diabetes with insulin-producing cells derived in vitro from human pluripotent stem cells. Nat Biotechnol.

[7] Zhang D, Jiang W, Liu M, Sui X, Yin X, Chen S, Shi Y, Deng H (2009). Highly efficient differentiation of human ES cells and iPS cells into mature pancreatic insulin-producing cells. Cell Res.

[8] Offield MF, Jetton TL, Labosky PA, Ray M, Stein RW, Magnuson MA, Hogan BL, Wright CV (1996). PDX-1 is required for pancreatic outgrowth and differentiation of the rostral duodenum. Development.

[9] Schaffer AE, Freude KK, Nelson SB, Sander M (2010). Nkx6 transcription factors and Ptf1a function as antagonistic lineage determinants in multipotent pancreatic progenitors. Dev Cell.

[10] Basford CL, Prentice KJ, Hardy AB, Sarangi F, Micallef SJ, Li X, Guo Q, Elefanty AG, Stanley EG, Keller G (2012). The functional and molecular characterisation of human embryonic stem cell-derived insulin-positive cells compared with adult pancreatic beta cells. Diabetologia.

[11] Sander M, Sussel L, Conners J, Scheel D, Kalamaras J, Dela Cruz F, Schwitzgebel V, Hayes-Jordan A, German M (2000). Homeobox gene Nkx6.1 lies downstream of Nkx2.2 in the major pathway of beta-cell formation in the pancreas. Development.

[12] Walczak MP, Drozd AM, Stoczynska-Fidelus E, Rieske P, Grzela DP (2016). Directed differentiation of human iPSC into insulin producing cells is improved by induced expression of PDX1 and NKX6**.**1 factors in IPC progenitors. J Transl Med.

[13] Goparaju SK, Kohda K, Ibata K, Soma A, Nakatake Y, Akiyama T, Wakabayashi S, Matsushita M, Sakota M, Kimura H (2017). Rapid differentiation of human pluripotent stem cells into functional neurons by mRNAs encoding transcription factors. Sci Rep.

[14] Akiyama T, Wakabayashi S, Soma A, Sato S, Nakatake Y, Oda M, Murakami M, Sakota M, Chikazawa-Nohtomi N, Ko SB (2016). Transient ectopic expression of the histone demethylase JMJD3 accelerates the differentiation of human pluripotent stem cells. Development.

[15] Hirayama M, Ko SBH, Kawakita T, Akiyama T, Goparaju SK, Soma A, Nakatake Y, Sakota M, Chikazawa-Nohtomi N, Shimmura S (2017). Identification of transcription factors that promote the differentiation of human pluripotent stem cells into lacrimal gland epithelium-like cells. NPJ Aging Mech Dis.

[16] Akiyama T, Wakabayashi S, Soma A, Sato S, Nakatake Y, Oda M, Murakami M, Sakota M, Chikazawa-Nohtomi N, Ko SBH (2017). Epigenetic manipulation facilitates the generation of skeletal muscle cells from pluripotent stem cells. Stem Cells Int.

[17] Akiyama T, Sato S, Chikazawa-Nohtomi N, Soma A, Kimura H, Wakabayashi S, Ko SBH, Ko MSH (2018). Efficient differentiation of human pluripotent stem cells into skeletal muscle cells by combining RNA-based MYOD1-expression and POU5F1-silencing. Sci Rep.

[18] Akutsu H, Machida M, Kanzaki S, Sugawara T, Ohkura T, Nakamura N, Yamazaki-Inoue M, Miura T, Vemuri MC, Rao MS (2015). Xenogeneic-free defined conditions for derivation and expansion of human embryonic stem cells with mesenchymal stem cells. Regen Ther.

[19] Warren L, Manos PD, Ahfeldt T, Loh YH, Li H, Lau F, Ebina W, Mandal PK, Smith ZD, Meissner A (2010). Highly efficient reprogramming to pluripotency and directed differentiation of human cells with synthetic modified mRNA. Cell Stem Cell.

[20] Nostro MC, Sarangi F, Yang C, Holland A, Elefanty AG, Stanley EG, Greiner DL, Keller G (2015). Efficient generation of NKX6-1+ pancreatic progenitors from multiple human pluripotent stem cell lines. Stem Cell Reports.

